# The Protective Effect of Ginsenoside Rg1 on Apoptosis in Human Ankle Joint Traumatic Arthritis Chondrocytes

**DOI:** 10.1155/2022/6798377

**Published:** 2022-04-21

**Authors:** Zhiqiang Xu, Xue Li, Guodong Shen, Yunxuan Zou, Hongning Zhang, Kangyong Yang, Yongzhan Zhu

**Affiliations:** ^1^Orthopaedics Center, Foshan Hospital of Traditional Chinese Medicine, Guangzhou University of Chinese Medicine, Foshan 528000, China; ^2^8th Department of Orthopaedics, Foshan Hospital of Traditional Chinese Medicine, Guangzhou University of Chinese Medicine, Foshan 528000, China

## Abstract

The ankle biomechanics is easily changed due to the acute injury of the tissue around the ankle joint and the damage of the ankle joint structure, such as ankle instability and joint surface imbalance. When the mechanical load of the ankle changes, it can cause ankle regeneration and remodeling processes such as cartilage loss, bone remodeling, and degenerative changes. The aim of this study was to investigate the effect and mechanism of ginsenoside Rg1 against interleukin-1*β* (IL-1*β*)-induced apoptosis in human articular chondrocytes (HACs). The apoptosis model of HAC cells was established by IL-1*β* induction, and then the HAC cells were cultured with different concentrations of Rg1. The protective effect of Rg1 on HAC cell apoptosis was investigated by detecting the changes of apoptosis and activity of PI3K/Akt/mitochondrial signaling pathway. The results showed that a specific concentration of Rg1 could promote the proliferation of IL-1*β*-induced HAC cells and inhibit apoptosis. At the same time, Rg1 treatment with specific concentration can reduce the content of reactive oxygen species (ROS) and malondialdehyde (MDA) in HACs and improve the related expression of mitochondrial membrane potential (MMP). Furthermore, qRT-PCR and western blot results showed that Rg1 could improve the low expression of Bcl-2 and inhibit the high expression of Bax, caspase-3, caspase-8, caspase-9, FasL, AIF, and Cyto c in IL-1*β*-induced cells. In summary, Rg1 can inhibit IL-1*β*-induced apoptosis of HAC cells by decreasing the activity of PI3K/Akt/mitochondrial signaling pathway, and Rg1 has a protective effect on apoptosis of HAC cells.

## 1. Introduction

Traumatic arthritis is followed by joint trauma; clinical pain and dysfunction signs often lag behind the initial injury for years or decades, accounting for about 12% of all types of osteoarthritis (OA) [1]. Ankle sprains are the most common sports-related injuries, involving the lateral collateral ligament complex in 85% of cases [2]. Any trauma to damage the surface of ankle can lead to the occurrence of ankle traumatic arthritis; the most common traumatic causes are considered to be intra-ankle fractures resulting in cartilage damage and ligament instability [3–5]. Apoptosis is considered to be one of the main causes of the loss of joint cartilage cells [6]. Apoptosis is designed to maintain environmental stability in the individual body, a process of independent and orderly cell death that is controlled by genes, regulated by a variety of cytokines and signaling pathways [7].

Cartilage protective drugs, which are nonsteroidal anti-inflammatory drugs, are the main drugs used to treat traumatic arthritis of human ankle joints [8, 9]. But their clinical effect of preventing or improving OA disease is not obvious [10]. Chinese medicine gained popularity in recent years for its potential therapeutic effects and low side effects [11, 12]. At present, ginseng saponin has been shown to have antagonistic apoptosis in many cells [13]. Gong et al. have found that ginsenoside Rg1 protected *β*-amyloid-induced apoptosis of primary cultured rat hippocampal neurons by increasing the Bcl-2/Bax ratio and inhibiting caspase-3 activation [14]. Hashimoto et al. then reported that ginseng saponins can inhibit the activation of PC12 cell line caspase-3 by activating the Akt and ERK1/2 signaling pathways and ultimately inhibit its apoptosis [15]. It can be seen that Rg1 does inhibit apoptosis, thus protecting related cells. In recent years, ginsenoside Rg1 has also been studied in osteoarthritis. Rg1 can treat both osteoarthritis and anterior cruciate ligament transection in rats. Rg1 can inhibit the inflammatory response of chondrocytes in vitro and reduce articular cartilage damage in rats. Rg1 has good research significance in the treatment of osteoarthritis. However, the mechanism of Rg1 in the treatment of osteoarthritis needs further study.

Mitochondria are susceptible parts of various damage factors, and the change of mitochondrial membrane permeability is a key step in the survival process of cells [16]. Caspase is an evolutionarily conservative family of cysteine protease, and the signaling pathway of relying on caspase is the primary route of apoptosis [17, 18]. We suspect that Rg1 may inhibit the apoptosis of human articular chondrocytes (HACs) by affecting the PI3K/Akt/mitochondrial signaling pathway, ultimately reducing the production of inflammatory factors.

In this study, the IL-1 *β*-induced HAC apoptosis model was used to determine the protective effect of Rg1 on HAC apoptosis through PI3K/Akt/mitochondrial signaling pathway.

## 2. Materials and Methods

### 2.1. Culture and Identification of HAC

The knee cartilage of healthy volunteers was cut under sterile conditions. The knee cartilage was cut into 0.5–1 mm^3^ particles on a super-clean workbench. It was digested about 2 hours with trypsin and washed twice with D-Hanks solution [19]. Then, the 10× cartilage volume of 0.2% II-type collagen enzyme was added to digest the cartilage overnight. The next day, the raw fluid was removed by centrifuge to obtain the cells and the media were added. The cells were moved into 100 mm cell culture dish and incubated at 37°C. The fluid was changed 2 to 3 times a week. The cells were digested 3 min with 0.05% trypsin containing EDTA when it near fusion. The cells were subcultured for 3-4 generations to obtain the human articular chondrocytes (HACs). All volunteers signed informed consent before surgery. Meanwhile, the study has been approved by the Ethics Committee of Foshan City Hospital of the Guangzhou University of Chinese Medicine.

### 2.2. Immunofluorescence Detection

HAC cells were inoculated in Petri dishes with cover glass slides for further subculture. After the cells developed into a monolayer, the cover glass was removed and washed twice with PBS buffer. 4% paraformaldehyde was added and fixed for 4 h and then washed for 3 times with PBS. Sealing solution was added and sealed for 30 min and then washed with PBS for 3 times. The anti-collagen II antibody (GB14073; Servicebio, Wuhan, China) was added at the dilution of 1 : 300 and incubated overnight and then washed with PBST for 3 times. Cy3-labeled secondary antibody (GB21401; Servicebio, Wuhan, China) was added at the dilution of 1 : 500 and incubated at room temperature for 1 h without light and then rinsed with PBST for 3 times. Fluorescence microscopy was performed, and the luminescence was excited at 570 nm.

### 2.3. CCK-8 Assay

HACs were grown in 96-well microplates. The CCK-8 solution (PH687; DOJINDO, Japan) was then added to the medium and incubated at 37°C for 4 h. Cell viability was measured using Multiskan FC (Thermo Scientific, USA).

### 2.4. Flow Cytometry

Annexin V-FITC/PI (KL602, DOJINDO, Japan) staining was used to determine the number of apoptotic cells. In simple terms, 5 *μ*L PI and 10 *μ*L annexin V-FITC solutions were added to 200 *μ*L binding buffer, followed by cells resuspension and reaction for 10 min at 25°C in the dark. The apoptosis cells were analyzed using flow cytometry (BD, USA).

### 2.5. Reactive Oxygen Species (ROS)

HAC cells were added with different concentrations of Rg1 solution and incubated in a cell incubator at 37°C in the dark. The collected cells were added with trypsin 10 *μ*L and 1 mL PBS buffer and incubated. The cells were centrifuged at 4600*g* for 5 min. The supernatant was taken and centrifuged at 4,100*g* for 10 min. The supernatant was discarded, the precipitation was collected, and 200 *μ*L PBS was added to resuspend the mitochondrial extract. The instructions of the ROS test kit (BB-47051; BestBio, China) were followed. An appropriate amount of DCFH-DA solution was added to the mitochondria suspension and then incubated at 37°C in darkness for 15 min. The excitation wavelength was set at 488 nm, and the emission wavelength was set at 525 nm. The fluorescence intensity of ROS was measured using a fluorescence spectrophotometer.

### 2.6. Malondialdehyde (MDA) Activity

HAC cells were collected and evaluated for MDA activity using a commercial ELISA kit (MSK, Wuhan). The blank control well was set. The 50 *μ*L sample was taken out and added into the sample well. 50 *μ*L detection antibody was added, and the reaction well was sealed with a sealing plate membrane and incubated in an incubator at 37°C for 2 h. The reaction solution was disposed, and 300 *μ*L washing solution was added, washed 5 times repeatedly. Substrates A and B 50 *μ*L were added to each well and incubated at 37°C for 15 min in the dark. The 50 *μ*L stop solution was added and shook well. The OD value at 450 nm was determined by using an enzyme plate analyzer.

### 2.7. Mitochondrial Membrane Potential (MMP) Assay

The MMP kit (Beyotime, Haimen, China) was used to detect MMP in cells. HAC cells in 6-well plates were routinely cultured, washed with PBS, and resuspended. The cells were cultured in 500 *μ*L JC-1 working solution at 37°C for 20 min and washed with PBS twice. MMP ratios of cells were analyzed using a flow cytometer system (BD, USA).

### 2.8. qRT-PCR

The mRNA expression of gene was detected by RT-PCR. The total RNA was extracted by using the Total RNA Extraction Kit (TIANGEN, Beijing, China) and then reversely transcribed into cDNA. The corresponding reaction system was configured to conduct PCR on cDNA. The reaction conditions were as follows: preheating at 95°C for 3 min, 95°C for 1 min, 60°C for 30 seconds, 72°C for 1 min, a total of 35 cycles.

### 2.9. Western Blot

Cells were collected and cultured in cell culture plates. Total proteins were extracted from the cells for gel electrophoresis and membrane transfer. The target protein was detected by anti-Cyto c (1 : 1000), caspase-9 (1 : 1000), Bcl-2 (1 : 500), and FasL (1 : 1000) (Abcam, USA) antibodies. HRP-labeled secondary antibody (1 : 1000; Santa Cruz, USA) was combined with primary antibody and cultured at 25°C for 1 h. The bands were detected using an infrared imaging system (LI-COR Biosciences, Nebraska, USA).

### 2.10. Statistical Analysis

GraphPad 8.0 software was used to analyze the data, and the mean ± standard deviation was used for all analyses. ANOVA was used to analyze the differences between groups, with *P* < 0.05 regarded as significant. All experiments were repeated three times.

## 3. Results

### 3.1. Culture and Identification of HAC

Primary cells generally adhered early and gradually extended to the surrounding after adherence, tiling into a polygon or short shuttle shape (Figure 1(a)). After cultivating for about 1 week, 80% of the cells were nearly confluent, at which time they could be digested and passaged. The shape of the third-generation cells was similar to the primary cells, evenly distributed (Figure 1(b)) and can produce cartilage-specific matrix, which was conducive to the maintenance and recovery of chondrocyte phenotype (Figure 1(c)). The expression of collagen type 2 in HAC cells was observed by immunofluorescence assay, and the cells were cultured well (Figure 1(d)).

### 3.2. Rg1 Promotes the Proliferation of HAC

There was no significant difference between the groups at 24 h (*P* > 0.05), and there was significant difference in cell proliferation promotion between the groups at 48 h and 72 h (Figure 2). Moreover, the high dose of Rg1 (100 *μ*g/mL) exhibited an increase in cell viability between the groups at 48 h and 72 h. This indicates that the appropriate concentration of Rg1 obviously promotes the proliferation of HAC, and the high concentration of Rg1 obviously promote the cell proliferation with the culturing time.

### 3.3. Rg1 Inhibits Apoptosis of IL-1*β*-Induced HAC

We used the culture of IL-1*β* (10 *μ*g/L) as an experimental concentration to induce HAC for 24 h and then treated the HAC with different concentrations of Rg1.  Figure 3 shows the result of HAC being tested by a flow cytometer. The rate of apoptosis cells in the IL-1*β*+0 *μ*g/mL Rg1 group was significantly higher than that of the control group (*P* < 0.05). The apoptosis rate of Rg1 treatment group was markedly lower than that of the IL-1*β* group and was in a concentration-dependent manner.

### 3.4. Effect of Rg1 on HAC Cell Mitochondrial Signaling Pathways

In order to further clarify the protective effect of Rg1 on mitochondrial apoptosis, we detected the levels of ROS and MDA in cells of different treatment groups. The results of the fluorescence spectrophotometer showed that the ROS content in IL-1*β*-induced cells was significantly increased (*P* < 0.001). The ROS contents in the IL-1*β*+(10, 50, 100 *μ*g/mL Rg1) groups were significantly lower than that in the IL-1*β* group (Figure 4(a)). In addition, the MMP test results showed that the MMP was significantly decreased in the IL-1*β* group, but the inhibition was reversed with the increase of Rg1 concentration (Figure 4(b)). The results showed that MDA content in IL-1*β* -induced cells was significantly increased, and increased Rg1 concentration could effectively reduce MDA content in IL-1*β* -induced cells (Figure 4(c)). To further explore how Rg1 inhibits mitochondrial pathway apoptosis, qRT-PCR and western blot analysis showed that IL-1*β-*induced cells reduced Bcl-2 expression and increased the expression of Bax, caspase-3, caspase-8, caspase-9, FasL, AIF, and Cyto c expressions (all *P* < 0.01) (Figures 4(d) and 4(e)). Mitochondrial apoptosis induced by IL-1*β* can be ameliorated by treatment with Rg1.

## 4. Discussion

Recent studies have found that Rg1 has a higher medicinal effect because of its antiapoptosis effect in a variety of cells. Gong et al. observed that in the neurons of the hippocampus, Rg1 has antagonistic amyloid-induced apoptosis, which can be used as a neuroprotector [14]. Yan et al.'s study found that Rg1 had a protective effect on *β*-amyloid-induced epithelial apoptosis [20]. In our present study, we found that the use of different concentrations of Rg1 pretreatment of HAC of IL-1*β* showed that the apoptosis rate of HAC was significantly lower than that of the IL-1*β* group, indicating that Rg1 did have an effect in suppressing HAC apoptosis.

The signaling pathway mechanism for the effect of Rg1 on the apoptosis of cartilage cells is not yet known. Studies have shown that blocking the PI3K/Akt/mitochondrial signaling pathway can reduce the apoptosis of IL-1*β*-induced cartilage cells in cartilage cells [21, 22]. Mitochondrial function plays an important role in the process of apoptosis [23]. Bcl-2 family protein is the main protein for mitochondrial pathways to regulate apoptosis, while Bcl-2 and Bax are the most representative inhibitory apoptosis and promoter proteins in the Bcl-2 family, respectively [24, 25]. Caspase-3 is the most important promoter of apoptosis, downstream of the apoptosis-affiliated reaction, resulting in cell death [26]. The Fas/FasL system is one of the leading signal transduction pathways for mediated apoptosis. Most cell procedural deaths are involved in the Fas/FasL system [27]. AIF is present in mitochondrial gap and can reduce the damage caused by oxidation stress to cell membranes and DNA by removing free radicals in cells through the redox reaction, thereby preventing apoptosis and acting as anti-cell apoptosis [28]. In this study, ROS and MDA content in IL-1*β*-induced HAC cells were significantly reduced by Rg1 treatment at different concentrations. In addition, high concentrations of Rg1 treatment increased the decrease of MMP in IL-1*β*-induced cells. Furthermore, qRT-PCR and western blot results showed that Rg1 increased the Bcl-2 downregulation and the expression of Bax, caspase-3, caspase-8, caspase-9, FasL, AIF, and Cyto c in IL-1*β*-induced cells. Huang et al. also confirmed that ginsenoside Rg1 can block caspase-3 release and protect rat chondrocytes from IL-1*β*-induced mitochondrial activated cell apoptosis through the PI3K/Akt signaling pathway [29]. This study is consistent with Huang's study that the PI3K/Akt signaling pathway plays a significant role in osteoarthritis. In the future, we can explore more treatments for osteoarthritis from the PI3K/Akt signaling pathway and mitochondrial activation pathway.

There are some shortcomings in our experiment. We have only conducted an in vitro experimental study of the effects of Rg1 inhibiting HAC apoptosis, and evidence of in vivo experiments is needed to further determine that Rg1 has inhibited HAC apoptosis.

## 5. Conclusion

In summary, we found that Rg1 may regulate IL-1*β*-induced HAC apoptosis through the PI3K/Akt/mitochondrial signaling pathway. Our results provide reliable evidence that Rg1 regulates the PI3K/Akt/mitochondrial signaling pathway in human ankle traumatic arthritis and strongly support Rg1 as a promising drug target for the treatment of ankle traumatic arthritis.

## Figures and Tables

**Figure 1:** Culture and identification of HAC. (a) The primary cells of HAC. (b) The third-generation cells of HAC. (c) The third-generation cells of HAC adherent growth (200×). (d) Detection of type 2 collagen in HAC by immunofluorescence.

**Figure 2:** Rg1 promotes the proliferation of HAC. The cell viability was evaluated by MTT assay (^*∗*^*p* < 0.05).

**Figure 3:** Rg1 inhibits apoptosis of IL-1*β*-induced HAC. After the chondrocytes were treated with IL-1*β* or different concentrations of Rg1, apoptosis was detected by flow cytometry (^*∗*^*p* < 0.05).

**Figure 4:** Effect of Rg1 on HAC cell mitochondrial signaling pathways. (a) The relative intensity of ROS was evaluated by cellular immunofluorescence. (b) The variation of MMP was evaluated by JC-1. (c) The content of MDA was evaluated by ELISA assay. (d) The Bax, Bcl-2, caspase-3, caspase-8, caspase-9, FasL, AIF, and Cyto c mRNA expressions were evaluated by qRT-PCR. (e) The Bax, Bcl-2, caspase-3, caspase-8, caspase-9, FasL, AIF, and Cyto c protein expressions were evaluated by western blot. Values with different letters within the same column differ significantly (^*∗*^*p* < 0.05).

## Data Availability

The data used to support this research are included within this manuscript.
